# Design and Implementation of Human Motion Recognition Information Processing System Based on LSTM Recurrent Neural Network Algorithm

This article has been retracted.

**DOI:** 10.1155/2021/3669204

**Published:** 2021-07-06

**Authors:** Xue Li

**Affiliations:** Department of Physical Education, Xi'an International Studies University, Xi'an 710128, Shaanxi, China

## Abstract

With the comprehensive development of national fitness, men, women, young, and old in China have joined the ranks of fitness. In order to increase the understanding of human movement, many researches have designed a lot of software or hardware to realize the analysis of human movement state. However, the recognition efficiency of various systems or platforms is not high, and the reduction ability is poor, so the recognition information processing system based on LSTM recurrent neural network under deep learning is proposed to collect and recognize human motion data. The system realizes the collection, processing, recognition, storage, and display of human motion data by constructing a three-layer human motion recognition information processing system and introduces LSTM recurrent neural network to optimize the recognition efficiency of the system, simplify the recognition process, and reduce the data missing rate caused by dimension reduction. Finally, we use the known dataset to train the model and analyze the performance and application effect of the system through the actual motion state. The final results show that the performance of LSTM recurrent neural network is better than the traditional algorithm, the accuracy can reach 0.980, and the confusion matrix results show that the recognition of human motion by the system can reach 85 points to the greatest extent. The test shows that the system can recognize and process the human movement data well, which has great application significance for future physical education and daily physical exercise.

## 1. Introduction

With the development of information technology, information processing system became a common form of human-computer interaction, widely used in all walks of life, and an important tool for various fields to obtain and store information, so the current research on information processing system is also increasing [1]. Tan et al. proposed a reservoir computing (RC) scheme for parallel processing of Santa Fe time series prediction task and signal classification task, performed a numerical research on its performance, and found that it has a very small error [2]. Mai et al. proposed a pedestrian tracking and detection system, which combined convolutional neural network (CNN) and color information to locate the pedestrians in the video frame, and then assigned the detected pedestrians to the corresponding path according to the similarity of color distribution [3]. Singh et al. recently proposed a quantum communication model system suitable for future information and communication technology and methodology flow, showing how to use block chain in quantum computing and quantum cryptography to provide security and privacy in information sharing [4]. Chen proposed a comprehensive medical information system with security policy and privacy protection function, which can effectively apply and save medical resources, meet the mobility of medical records, and reflect the function and security of drug collection [5]. Tang and other scholars designed an improved hybrid algorithm under the deep learning of information technology and applied it to the actual medical material distribution system, which effectively reduced the distribution cost, shortened the transportation route, and improved the optimization efficiency [6]. Wang and Li combined OWA with grey correlation analysis to propose a mobile information retrieval system with higher recommendation effect [7].

Additionally, a large number of studies have been reported on neural network algorithms. Dong et al. studied the robust exponential stabilization of uncertain discrete-time stochastic neural networks with time-varying delays based on output feedback control [8]. Date et al. described an improved DNN based analysis method, using the mean reduced accuracy (MDA) calculation based on permutation algorithm to estimate the importance of each variable [9]. Yin et al. proposed a simple two-phase algorithm BinaryRelax, which is used to train deep neural networks with quantization weights. The set constraint of quantization weights is not imposed until the later stage of training [10]. Isik and other scholars used artificial neural network and fuzzy inference system based on adaptive network to model the data of General Administration of Meteorology (MGM) and model and predict the forward-looking data with high sensitivity in thermal system, with satisfactory results [11]. Wang et al. studied the global Mittag-Leffler stability of fractional order neural networks (FNNs) with piecewise constant arguments and finally verified the effectiveness of the results by an example [12]. Zazo et al. proposed a new age estimation system based on LSTM RNNs, which can handle short speech and can be easily deployed on a real-time architecture [13]. Cortez et al. proposed a new EV prediction architecture based on recurrent neural network (RNN). Through the evaluation of the historical data of electric vehicles provided by the Guatemalan national police, the effectiveness of this architecture compared with the traditional time series analysis and machine learning methods was demonstrated [14]. Bahad et al. proposed a false news detection model based on bidirectional LSTM recurrent neural network, and after testing and evaluation, it shows that, for false news detection, bidirectional LSTM model is superior to CNN, vanilla RNN, and unidirectional LSTM in accuracy [15].

To sum up, with the advent of the information age, experts and scholars all over the world are studying the information processing system. Simultaneously, many scholars analyzed the application of neural network, and some scholars combined the two to extract and process information. With the popularity of artificial intelligence and development of smart city, there is an urgent need for an algorithm mechanism that can quickly and accurately identify human behavior. The advantages of information processing system can also be reflected. However, there are few research reports on the use of information processing system to analyze human motion. Simultaneously, according to the analysis of neural network, it is found that LSTM recurrent neural network can well solve the problem of long-term dependence. Therefore, in response to the national fitness program of our country, this research will perform the design of human motion recognition information processing system based on LSTM recurrent neural network algorithm, hoping to build an intelligent sports ecosystem and promote the development of China's sports industry.

## 2. Theoretical Analysis of Human Motion Recognition Information Processing System Based on LSTM Algorithm

### 2.1. The Architecture of Identification Information Processing System

Human motion recognition system is a kind of computer software system that collects human motion data through sensors and other acquisition hardware and then uses related algorithms for data processing [16]. Similar to other processing systems, human motion information recognition is still related to data exchange, processing, and analysis. Therefore, according to other system architecture schemes, a human motion recognition information processing system is proposed, as shown in Figure 1.

Figure 1 shows that the proposed information processing system is divided into three layers, in which the data collection layer needs to use all kinds of motion sensors to collect human motion data, and then transmits the data to the preprocessing module to process the data into standard data. As the core layer of the system, the data computing layer is responsible for sorting out the preprocessed data and storing it in the database. However, it needs to further identify the preprocessed data. In this process, it will classify and store the data. The third layer is the level of user contact, which mainly includes user interface and data visualization. Users can clearly understand their own motion state through interface instructions.

Currently, the motion sensors on the market are mostly used in wearable sports devices and smart phones, which are mainly used to collect the acceleration, angular velocity, and location of human motion. In this study, three-week gyroscope, accelerometer, and magnetometer will be used to collect the previously mentioned three kinds of human motion data [17, 18].

There are two main tasks in the system data preprocessing, noise filtering and data normalization. In the noise filtering process, it mainly deals with the system noise in the human movement data and the data deviation caused by the sudden vibration of our school outside. Various noises are removed as much as possible by filtering. In addition, unnecessary missing values in the data need to be removed by deleting and other methods [19, 20]. The purpose of data normalization is to identify and compare the data of different dimensions at the same latitude. The transformation formula is shown as follows:

(1) $$\begin{array}{c} x^{\prime }=\frac{x-\min\left(x\right)}{\max\left(x\right)+\min\left(x\right)}, \end{array}$$

where min(*x*) and min(*x*) represent the data values of the minimum and maximum values, respectively.

The calculation of data needs three stages. The first stage is to store the data. In the storage module, we need to build a core database. In addition, we need to segment the stored preprocessed data. The purpose is to extract the frequency domain features of the data more conveniently. The segmented data is input to the feature extraction module for data recognition and classification. The features to be extracted include the mean value, and the calculation formula is shown as follows:

(2) $$\begin{array}{c} \text{mean}=\underset{n⟶\infty }{\lim}\frac{1}{n}\sum_{i=1}^{n}\alpha_{i}, \end{array}$$

where mean is the mean value and *α*_*i*_ is the *i* − th data value. The calculation method of standard deviation is shown as follows:

(3) $$\begin{array}{c} \text{std}=\underset{n⟶\infty }{\lim}\sqrt{\frac{1}{n}\sum_{i=1}^{n}{\left(\alpha_{i}-\text{mean}\right)}^{2}}, \end{array}$$

where std is the standard deviation of data and mean is the average of all data. The calculation method of the maximum value is shown as follows:

(4) $$\begin{array}{c} \max=\max\left(\alpha_{i}\right),\;i\in \left\{1,2,3,\ldots \right\}, \end{array}$$

where max is the maximum value in the data and *i* represents the total number of data. Similarly, the minimum value is calculated as follows:

(5) $$\begin{array}{c} \min=\min\left(\alpha_{i}\right),\;i\in \left\{1,2,3,\ldots \right\}, \end{array}$$

where minis the maximum value in the data. In addition, the signal amplitude area of the data information needs to be solved as follows:

(6) $$\begin{array}{c} \text{SMA}=\frac{1}{t}\int_{0}^{t}\left|z\left(t\right)\right|\text{d}t, \end{array}$$

where *z*(·) is the signal curve and *t* is the time. The calculation formula of data signal skewness is shown as follows:

(7) $$\begin{array}{c} SK=\frac{\underset{n⟶\infty }{\lim}\left(1/n\right)\sum_{i=1}^{n}{\left(x_{i}-\bar{x}\right)}^{3}}{\underset{n⟶\infty }{\lim}{\left[\left(1/n\right)\sum_{i=1}^{n}{\left(x_{i}-\bar{x}\right)}^{2}\right]}^{3/2}}, \end{array}$$

where *x*_*i*_ is the *i*_th data and $\bar{x}$ is the average value. Finally, the abundance of the data curve is calculated as follows:

(8) $$\begin{array}{c} K=\frac{\underset{n⟶\infty }{\lim}\left(1/n\right)\sum_{i=1}^{n}{\left(x_{i}-\bar{x}\right)}^{4}}{\underset{n⟶\infty }{\lim}{\left[\left(1/n\right)\sum_{i=1}^{n}{\left(x_{i}-\bar{x}\right)}^{2}\right]}^{2}}. \end{array}$$

where *K* stands for kurtosis, which is mainly used to compare the extreme and average values of the curve, so as to judge whether the curve is smooth or not.

### 2.2. LSTM Recurrent Neural Network

LSTM recurrent neural network is a long-term and short-term memory network, which is proposed to solve the long-term dependence problem in traditional recurrent neural network. LSTM recurrent neural network is a nonlinear model, which can be used in continuous recognition without segmentation. This is one of the reasons why this network is selected in this study, which is to ensure continuous recognition in the process of human movement and theaccuracy of the data. LSTM recurrent neural network adds many gates and memory units to the traditional recurrent neural network, and the schematic diagram is shown in Figure 2.

As shown in Figure 2, three gates are added to the LSTM unit, namely, forgetting gate *f*_*t*_, input gate *i*_*t*_, and output gate *h*_*t*_. The function of forgetting gate is to output the last moment, according to the current output to determine the forgetting part of the memory. The function of output gate is also to filter out unnecessary information, so as to determine that part of the information can enter the neural unit. The memory unit in LSTM neural network is affected by input gate and forgetting gate, and the state of memory unit depends on the state of the last memory unit. Finally, the memory unit controls the data output of the neural unit, thus controlling the data output degree of the output gate. The expression of the excitation function in the neural network is shown as follows

(9) $$\begin{array}{c} \sigma \left(x\right)=\frac{1}{1+\sigma^{-x}}, \end{array}$$

where *σ*(*x*) represents the excitation function, which is mainly responsible for the nonlinear transformation of the linear output in the network. It is the simulation diversification of neural network and can simulate the nonlinear function.

For the layer number design of neural network, the general neural network design method is adopted, and three network layers are set, namely, input layer, hidden layer, and output layer. In this study, softmax function is selected as the excitation function of full connection layer [21, 22]. Additionally, the choice of the loss function determines the prediction performance of the model:

(10) $$\begin{array}{c} L_{i}=-\sum_{j}t_{i,j}\log\left(p_{i,j}\right), \end{array}$$

where *p* is the predicted value, *t* is the actual data value, *i* is the actual data, and *j* is the classification of the data displayed in the prediction. To minimize the loss of function and achieve accurate fitting, gradient descent algorithm is added to the model to iteratively optimize the loss of function and finally calculate the optimal solution:

(11) $$\begin{array}{c} \theta =\theta -\alpha \cdot \frac{\partial_{J}\left(\theta \right)}{\partial \theta }, \end{array}$$

where *α* represents the learning rate, which is mainly used to control the speed of the whole model during training. Then, it represents the gradient of the function. The function calculates the sample size required by the gradient and uses the small batch gradient descent algorithm to calculate. Each iteration only samples a small batch of samples, so as to improve the accuracy and efficiency of the algorithm.

## 3. Structure Design of Human Motion Recognition Information Processing System

### 3.1. System Structure and Function Analysis

The human motion recognition information processing system mainly collects a large amount of motion data with the help of the relevant equipment installed with sensors, identifies the daily motion data of users, stores the data, and visualizes the time in the human-computer interaction interface of the system, so that users can view personal motion files in real time [23]. It should be noted that if we want to get more accurate human motion data, we need to refer to a large number of human motion information. This study uses LSTM neural network model to process and identify a large number of human motion data. For example, the system proposed in the study is divided into three modules, namely, data acquisition module, data calculation module, and data application module. The three modules work together to realize the system function, as shown in Figure 3.

As shown in Figure 3, the system structure based on LSTM recurrent neural network includes three modules. The functions of the three modules need to realize the recognition and classification of human movement information data. The means of recognition and classification is to use data mining technology to classify the sports data collected by wearable devices. In addition, the visualization function of the system is to draw a visual analysis view of the uploaded movement data in three-dimensional mode, and the user information management function is to manage and store the user's personal account information and physical characteristics, so as to facilitate the association of user movement data. The user's movement data management is the function of the system to manage the user's movement state and movement state changes or other movement data. It can be combined with the user information management function to help users understand their own movement situation more clearly and predict the user's future movement trend.

### 3.2. Design of Information Processing System

The data recognition effect of the system is directly determined by the performance of the model, and the performance of the model needs a large number of data under multiple factors for training. For personal movement data, the external data to be collected should be the diversified data of gender, age, and body shape. To train the model, the dataset used in this experiment is based on the human movement data published by a large number of researchers on the Internet to form the final model, which is conducive to reflecting the accuracy of LSTM circular neural network model [24, 25]. The data calculation and classification of the system is mainly to calculate, classify, and store user information, motion types, motion data, and model files. The data segmentation of the system needs to use sliding window to process data. This research designs a sliding window with a width of 200 according to the actual human movement, and the moving step of the designed window is 100. This design can fully accommodate a complete action and will not reduce the recognition accuracy due to the excessive width of the window. Finally, the algorithm module of LSTM recurrent neural network is constructed, as shown in Figure 4.

As shown in Figure 4, the model framework contains input, LSTM, and output layers. *X*, *Y*, and *Z* in the output layer are buffers. The data collected by the collector from the user is a kind of three-dimensional vector, and the data is sent to LSTM layer for data preprocessing. It can be found that only two layers of LSTM are designed in the hidden layer. The number of nodes in the first layer is 128, and the number of nodes in the second layer is 12. The purpose is to ensure that the model does not over fit. The output layer of the model uses softmax as the incentive function and uses the mechanism of full connection layer to realize the classification output of data.

The more important part of the system is the data application layer, that is, the user interface of the system. A good user interface can improve the user's interaction experience, including the system entrance, which is mainly used to determine whether the user is authorized to log in. Then, the interface of the system, including the home page and user interface, can visualize the user's motion data and can push the user's motion data recognized by the system.

## 4. Practical Application and Test Results of Human Motion Information Recognition System

### 4.1. Analysis of Training Results of LSTM Recurrent Neural Network Model

The dataset used in this experiment is the standard open dataset pamap2, which is proposed by the University of California, and contains a large number of body movement data. In this experiment, 80% of the dataset is used as the training set, and the remaining 20% is used as the test set of the model. The training results are shown in Figure 5.

As can be seen from Figure 5, when the model has been trained for 20 iterations, the accuracy of the model begins to gradually flatten. At this time, the system loss value still has a certain degree of downward trend. When the number of iterations reaches 100, the accuracy and loss value of the model begin to stabilize. The experiment found that if the number of LSTM layers is increased, the accuracy of the model will be improved to a certain extent, but it also increases the training time of the model, so according to the experimental results, the number of two layers LSTM used in the study is more appropriate. The trained model is compared with other models. The algorithms used in this comparison are rotation forest, K-NN. and BP-NN [26]. The advantages and disadvantages of LSTM neural network model are analyzed. The results are shown in Figure 6.

As can be seen from Figure 6, in the test analysis using the same dataset, the BP-NN algorithm with the lowest accuracy is 0.972, followed by the KNN algorithm with the accuracy of 0.977. The accuracy of LSTM algorithm can reach 0.980. Additionally, the accuracy of LSTM algorithm is similar to that of rotation forest algorithm, but the accuracy of LSTM algorithm is still higher than that of rotation forest algorithm. The previously mentioned results show that the accuracy of LSTM neural network algorithm is higher, and it is significantly better than other traditional algorithms. The reason for this is that LSTM has a special memory ability compared with other traditional algorithms, so it can make better prediction and analysis for the next step according to the current information when identifying the data. After testing, the confusion matrix of LSTM recurrent neural network model is generated as shown in Figure 7.

It can be seen from Figure 7 that LSTM model can well classify most of the motion categories, and according to the results of confusion matrix, the model gives a more positive value for most of the motion categories. However, it is not difficult to see that the model is still not very accurate in judging some confusing movements, such as the two movements of going downstairs and going upstairs. The reason is that the movement data and postures of the people going upstairs and downstairs are roughly similar, and the model needs to continue deep learning to fully distinguish the two movements to achieve more accurate judgment.

### 4.2. Application Effect of Human Motion Information Recognition System

The development environment of the system is Intel quad core CPU, 3.2 GHz, 1000 g hard disk, and 12 g memory. It is written by Python in ubuntu16.04 system. Two computers are used in the system test, wearable devices are configured on the subjects, the system interface is opened in the web page, and the subjects are instructed to start running. The movement data are shown in Figure 8.

As can be seen from Figure 8, the system recognizes the acceleration, angular velocity, and geomagnetism of the subject in running state, and the motion data transmitted from different sensors can be clearly displayed in the curve. In addition, the movement state recognition results of the subjects by the observation system show that the largest judgment value is running, followed by cycling, but the system displays according to the total judgment value and finally determines that the subject's current movement state is running state. The previously mentioned results show that the system can recognize human motion data quickly and judge human motion state according to multiple sensors, and the accuracy is very high.

In addition to better reflect the recognition effect of the system for different types of motion states, the recognition results of different types of motion are compared and analyzed to find the recognition characteristics and rules in the system, as shown in Figure 9.

Figure 9 shows the comparison results of the motion data of sitting and lying in two motion states. It can be seen from Figure 9 that the curve fluctuation of the two motion states is not obvious and the fluctuation speed of each sensor is almost 0, because sitting and lying are not periodic motion, so the data change of the human body in the two motion states will only show a certain instantaneous fluctuation. However, it can be seen that, despite this, the system can well distinguish the two kinds of motion states, mainly in the difference of geomagnetic values under the two kinds of motion states. Due to the different body position changes under the two kinds of motion states of sitting and lying, there will be differences in the direction of body changes. Simultaneously, other motion states identified in the system are compared, as shown in Figure 10.

In Figure 10, we compared the movement data curves of cycling and going upstairs. It can be seen from the motion data of cycling and going upstairs that the data curve of cycling shows that the difference between the peak and trough of acceleration is small, and the fluctuation is not obvious. On the contrary, in the action of going upstairs, the human body needs to overcome the gravity, which leads to a great instantaneous extreme value of acceleration. The system judges the state of human movement according to some of the differences. According to the previously mentioned comparison results, it can be clearly seen that the system designed in this study has a strong ability of recognition and classification. In addition to the daily movement of human body, some other sports data are analyzed in the experiment to analyze the universality of LSTM information processing system. The experimental results are shown in Figure 11.

Figure 11 shows that the system recognizes the subjects' actions as the foot slip and the center of gravity are not falling, and the actual subjects are in the two motion states. It can be seen that the motion of the foot slide is periodic transformation, and the amplitude of the step is different in different time periods. The data from each sensor shows that most of the fluctuation speed exceeds 100, but the fluctuation of the gravity center is not decreased. The results show that the system can recognize the motion data completely, which is very helpful for the practical teaching in the future.

## 5. Conclusion

In the face of the rapid development of science and technology and the upgrading of people's demand for life, people's attention to their own health is also rising, so the emergence of intelligent detection devices can help people to move. In this study, a recognition information processing system based on LSTM recurrent neural network is proposed to fill the vacancy of human motion data recognition and detection in the market. The human body data can be collected, processed, classified, and identified through the three-tier processing module in the system, and the data can be visualized in the user interface through the application layer. The main core of this system is the LSTM recurrent neural network. With the recognition ability and information feature processing ability of the neural network, the collected human motion data can be well analyzed and processed. According to the final experimental results, the data analysis ability of LSTM model is significantly better than other traditional algorithms, and the training accuracy can reach 0.983. From the test and analysis of practical application, it can be found that the effect of the system in human motion state recognition is excellent, and for similar motion state, the system can accurately determine according to the subtle data differences collected by the sensor. To sum up, for human motion data processing, using LSTM recurrent neural network for data feature extraction and recognition classification has a good effect, and the recognition process is relatively simple, to a certain extent, and increases the recognition efficiency of the system. The system will help assist sports training and can put forward corresponding suggestions for the actual sports.

## Figures and Tables

**Figure 1:** Human motion recognition information processing system.

**Figure 2:** Schematic diagram of LSTM recurrent neural network unit.

**Figure 3:** System structure and function.

**Figure 4:** Algorithm module of LSTM recurrent neural network.

**Figure 5:** Training results of LSTM recurrent neural network.

**Figure 6:** Comparison of recognition accuracy of multiple algorithms.

**Figure 7:** Confusion matrix of test data.

**Figure 8:** Motion data and recognition results.

**Figure 9:** Data chart of sitting and lying. (a) Sit and stand. (b) Lie.

**Figure 10:** Comparison of motion data in different motion states. (a) Cycling. (b) Go upstairs.

**Figure 11:** System identification results. (a) Foot slide. (b) The center of gravity does not drop.

## Data Availability

The data used to support the findings of this study are available from the corresponding author upon request.
